# Angelica sinensis Polysaccharide Alleviates Myocardial Fibrosis and Oxidative Stress in the Heart of Hypertensive Rats

**DOI:** 10.1155/2021/6710006

**Published:** 2021-09-03

**Authors:** Xiaolong Song, Junhong Kong, Jun Song, Renyou Pan, Lei Wang

**Affiliations:** ^1^Department of Cardiology, Yancheng Traditional Chinese Medicine Hospital Affiliated to Nanjing University of Chinese Medicine, Yancheng, Jiangsu Province, China; ^2^Department of Treating Disease Center, Changzhou Traditional Chinese Medicine Hospital Affiliated to Nanjing University of Chinese Medicine, Changzhou, Jiangsu Province, China; ^3^Laboratory of Morphology, Xuzhou Medical University, Xuzhou, Jiangsu Province, China

## Abstract

This research is aimed at studying the effect of Angelica sinensis polysaccharide (ASP) extracted from the Lixinshui prescription on cardiac disease induced by hypertension in rats. Rat models of cardiovascular disease were established, and the associated factors were measured. The data showed that ASP treatment increased the ejection fraction and short axis shortening rate, while decreasing the LV end-diastolic diameter, LV end-systolic diameter, LV end-diastolic volume, and LV end-systolic volume in HHD rats. ASP downregulated the expression level of TGF-*β*1, alpha-smooth muscle actin (*α*-SMA), collagen I, fibronectin, vimentin, Bax, cleaved caspase-9, and cleaved caspase-3 and upregulated the expression level of Bcl-2 in LV of HHD rats. Meanwhile, ASP increased the activity of superoxide dismutase (SOD) and glutathione peroxidase (GSH-Px) and decreased the level of malondialdehyde (MDA), tissue endogenous hydrogen peroxide (H_2_O_2_), and reactive oxygen species (ROS). Our findings indicated that ASP could prevent hypertensive heart disease by inhibiting myocardial fibrosis, suppressing the myocardial apoptosis, and alleviating oxidative stress.

## 1. Introduction

Cardiovascular diseases (CVDs) are the first cause of mortality and morbidity all around the word. Meanwhile, hypertension acts as the major risk factor in the cardiovascular disease development [1]. According to the estimate of the World Health Organization (WHO), the amount of hypertensive population worldwide will reach to 1.13 billion [2]. Hypertension often remains undiagnosed or untreated for a long time. However, hypertension may induce myocardium structural and functional changes. These changes include cardiomyocyte apoptosis, oxidative stress increase, and hypertrophy of the left ventricle. All of these can lead to the heart failure [3]. Nevertheless, even patients with hypertension have significantly higher hypertensive heart disease morbidity and mortality, and the effects of pharmacotherapy from current standard hypertension guidelines have unclear benefits on regression of left ventricular hypertrophy.

Recently, more and more traditional Chinese herbal medicines (TCMs) have been studied as the application for the treatment of cardiovascular diseases [4, 5]. For example, SINI Decoction (SND) is used to prevent and treat CVDs [6]. As one of the active components of Epimedium, icariside II improved left ventricular remodeling [7] and alleviated endoplasmic reticulum stress- (ERS-) induced cardiomyocyte apoptosis in spontaneously hypertensive rats (SHRs) [8]. The Lixinshui prescription was created by chief physician Zeng Xuewen to improve the cardiac function status of patients with chronic heart failure (heart edema syndrome). This prescription was studied to have a tendency to improve the ventricular remodeling [9]. The Lixinshui prescription is composed of ginseng, Radix Astragali, Yu Zhu, Gui Zhi, with tablets, Angelica, Chuanxiong, lepizi, and glossy ganoderma. Angelica sinensis polysaccharide (ASP) as the major bioactive component extracted from the roots of angelica exhibits beneficial antioxidation function in treating multiple diseases caused by oxidative stress [10, 11]. For instance, Wang and colleagues found that ASP attenuated liver injury in mice treated with concanavalin A [12]. The study of Cheng and colleagues showed that ASP promoted neurogenesis by enhancing the antioxidant and anti-inflammatory capacity and delayed aging speed by protecting neural stem cells (NSCs) [13]. However, the potential role of ASP in hypertension heart disease needs to be further explored.

In the current study, we established a hypertensive heart disease (HHD) rat model according to the previous study [14]. The potential effect of ASP extracted from the Lixinshui prescription on hypertensive heart disease was assessed by measuring various echocardiographic parameters of the left ventricle, examining the pathological features of cardiac tissues, investigating the expression of genes involved in fibrosis and apoptosis, and estimating the myocardial antioxidant status in left ventricle tissue. Our findings demonstrate that ASP, the active component of the Lixinshui prescription, is an excellent candidate for hypertensive heart disease. ASP could prevent hypertensive heart disease by inhibiting myocardial fibrosis, suppressing the myocardial apoptosis, and alleviating oxidative stress. These may facilitate the development of traditional Chinese herbs in modern medicine.

## 2. Material and Method

### 2.1. Plant Materials

The Lixinshui prescription was obtained from local Chinese medicine stores. The polysaccharide extraction and purification were performed as reported [12]. The molecular weight (MW) of ASP was 72.9 kD. The sugar content was approximately 95.1%, and there were no protein and nucleic acid detected in the content. Arabinose, glucose, and galactose were the constituent of ASP, and the molar ratio of the three monosaccharides was 1 : 2.5 : 7.5. Finally, the ASP was freeze-dried for storage.

### 2.2. Animal Experiments

This study was conducted with the consent from the Experimental Animals Ethics Committee. All procedures were carried out in accordance with the Guide for the Care and Use of Laboratory Animals.

Specific pathogen-free male Sprague-Dawley (SD) rats were used in this study. The rats were couple housed and maintained in a relative humidity (50 ± 20%) and temperature environment (25 ± 1°C) with a 12-hour light/dark cycle. All of the rats required a seven-day acclimation period before the experiment.

Twenty-four rats (weight 200-220 g) were induced to hypertensive heart disease (HHD) by an eight-week treatment with a high-fat diet (HFD) (standard diet added with 20% fat from lard, 20% sucrose, 10% protein, 1% cholesterol, and 0.5% sodium deoxycholate). After HHD 8-week treatment, the HHD rats were randomly divided into four treatment groups: three ASP-treated groups (80, 160, and 320 mg·kg^−1^ per day, respectively, named as LASP, MASP, and HASP) and one vehicle-treated group (model). The ASP was dissolved in distilled water and delivered through oral administration. The rats fed a common diet and orally administered distilled water (10 mL kg^−1^ per day) were set as the normal control group (control). All of the rats were allowed free access to the standard diet or high-fat diet during the experimental period.

### 2.3. Detection of Left Ventricular Function

The left ventricle function was measured as described [8] at the end of the experiment. Briefly, the rats were fixed on an animal operation platform after anesthesia. Then, various echocardiographic parameters were measured with a trimodal PET/SPECT/CT scanner. The parameters included left ventricle ejection fraction (EF), left ventricular short axis shortening rate (FS), left ventricle end-diastolic volume (LVEDV), left ventricle end-diastolic diameter (LVEDD), left ventricle end-systolic diameter (LVESD), and left ventricular end-systolic volume (LVESV). All results were calculated with the means of multiple consecutive cardiac cycles.

### 2.4. Measurement of Antioxidant Status

The left ventricle tissues of each rat (0.1 g) were added to 0.9 ml of sterile saline and fully homogenized. After centrifugation at 12,000 g for 10 minutes at 4°C, the supernatants of each group were gathered for further analysis. Five oxidative and antioxidative parameters including the activity of glutathione peroxidase (GSH-Px) and superoxide dismutase (SOD), the content of reactive oxygen species (ROS), endogenous hydrogen peroxide (H_2_O_2_), and malondialdehyde (MDA) were measured in the samples according to the details in the kit (Nanjing Jiancheng Bioengineering Institute, China).

### 2.5. Histological Examination

The rat left ventricle tissues were removed and fixed in formalin. Then, the tissues were washed with running water, dehydrated using graded ethanol (75%, 95%, 95%, 100%, and 100%), vitrified by xylene (twice), and embedded in paraffin wax. Next, the paraffin-embedded left ventricle tissue blocks were sectioned into 4 mm thick slides. The slides were deparaffinized by submersion in xylene, followed by rehydration with alcohol gradient (100%, 100%, 95%, 95%, and 75%). Finally, the slides were stained with H&E (C0105, Beyotime, China) or Masson's trichrome dye (G1340, Solarbio, China) to observe the pathological changes in left ventricle tissues under a microscope with 400x magnification. The areas of muscle fibers and myocardial fibrosis (red) or collagen (blue) were quantified using the ImageJ (National Institutes of Health, Bethesda, MD).

### 2.6. Immunofluorescence Assay

The rehydrated slides were restored with citrate antigen retrieval solution for 2 min by using a high-pressure steam boiler. Then, the slides were blocked in PBST solution (PBS added with 0.3% Triton X-100) with 1% BSA for 1 hour at room temperature. Next, the slides were incubated with *α*-SMA and TGF-*β*1 antibodies diluted in PBST solution with 1% BSA at 4°C overnight, respectively. FITC goat anti-rabbit IgG (ZSGB-Bio, China) was used as the secondary antibody and was diluted in PBST solution. The slides were incubated with the secondary antibody shielded from light for 1 hour, followed by staining with DAPI for another 10 minutes. Finally, the slides were imaged with a fluorescence microscope with 400x magnification.

### 2.7. TUNEL Staining

The rehydrated left ventricle tissue slides were assessed regarding the apoptosis activity with the Colorimetric TUNEL Apoptosis Assay Kit (C1098, Beyotime, China) according to the instructions. Briefly, the slides from each group were permeabilized with PBST on ice for 5 minutes and mixed with terminal deoxynucleotidyl transferase (TdT) enzyme for 2 hours, followed by reaction stop with PBST solution with 1% BSA for 10 minutes. Then, the slides were incubated with anti-digoxigenin-conjugated HRP for 30 and diaminobenzidine (DAB) solution for 20 minutes, subsequently. DAB reacts with the HRP-labelled sample to generate an insoluble colored (brown) substrate at the site of DNA fragmentation. The nuclei were counterstained with hematoxylin. Finally, TUNEL-positive cells were counted under a fluorescence microscope with 400x magnification. The percentage of apoptotic bodies = number of TUNEL‐positive cells/total number of cells × 100%.

### 2.8. Reverse Transcription Quantitative Polymerase Chain Reaction (RT-qPCR)

Total RNA was extracted from the left ventricle tissue according to the manual of TRIzol (Invitrogen, Carlsbad, CA, USA). cDNA was synthesized using PrimeScript RT Reagent (TaKaRa, Japan). The RT-qPCR was performed to detect the relative expression level of mRNA using a 7500 Real-Time PCR System (Applied Biosystems, Carlsbad, CA, USA). The primer sequences are listed in Table 1. The RT-qPCR analysis was performed using the 2^−ΔΔCT^ method.

### 2.9. Western Blotting

The left ventricle tissue homogenates were harvested in lysis buffer, put the samples on ice for 30 min, and collect the supernatant by centrifugation at 12,000 rpm at 4°C for 30 minutes. Protein concentration in the supernatant was measured by using the Enhanced BCA Protein Assay Kit (P0010S, Beyotime, China). 30 *μ*g of total proteins was separated on 12% sodium dodecyl sulfate polyacrylamide gel. Next, the proteins were electrically transferred onto PVDF membranes (Millipore). The membranes were incubated in PBST solution with 1% skim milk powder for 1 hour. Then, the membranes were incubated with antibodies specific to collagen I, *α*-SMA, fibronectin, vimentin, cleaved caspase-3, cleaved caspase-9, Bcl-2, and Bax at 4°C overnight. Meanwhile, *β*-actin was used as the standard control. The membranes were washed 4 times with PBST and incubated with the secondary antibody for another 1 hour. Finally, the protein bands were visualized with the incubated enhanced chemiluminescence system (ECL) for another 5 minutes. Protein levels were quantified using the ImageJ (National Institutes of Health, Bethesda, MD).

### 2.10. Statistical Analysis

GraphPad Prism (version 6.01 for Windows) statistical software was used to perform statistical analysis. The Student *t*-test was used to compare the significant differences between groups. ANOVA for repeated measures was used for intragroup analyses. Statistical significance was set at *p* < 0.01.

## 3. Results

### 3.1. Angelica sinensis Polysaccharide Improves Cardiac Function in Hypertensive Rats

Rats were fed an HFD for 8 weeks to induce hypertensive heart disease; then, the rats were orally administered either dose of ASP (80, 160, and 320 mg kg^−1^ per day) or distilled water over the last 6 weeks. The body weights of the HHD rats (model, LASP, MASP, and HASP groups) were significantly higher than the weights of normal rats (control group) during the experimental process. However, body weight of the HASP group rats in the final 6 weeks was lower than that of the model group rats (Figure 1(a)). Meanwhile, left ventricle function was measured before the rats were euthanized. The result showed that EF and FS were significantly decreased in the HHD rats in comparison with the normal rats. These indicated ventricular remodeling and dysfunction in the HHD rats. ASP significantly increased EF and FS in a dose-dependent manner in comparison with the model group rats (Figure 1(b)). At the same time, the LVEDD, LVESD, LVEDV, and LVESV were significantly increased in HHD rats in comparison with the normal rats; ASP significantly decreased LVEDD, LVESD, LVEDV, and LVESV in a dose-dependent manner compared with the model group rats (Figure 1(b)). All of these data indicated that ASP could recover cardiac dysfunction induced by hypertension in rats.

### 3.2. Angelica Polysaccharide Inhibits Cardiac Fibrosis in Hypertensive Rats

First, we performed H&E and Masson's trichrome staining to examine the effect of ASP on the histology of the hearts. The H&E-stained tissue slices showed that the hearts of normal rats had orderly, well-arranged myocardial cells. However, we observed disorderly arranged myocardial cells in HHD rats. And ASP significantly alleviated the disorderly arrangement in a dose-dependent manner in comparison with the model group rats. Meanwhile, Masson's trichrome-stained tissue slices showed that significantly thickened muscle fibers and significant myocardial fibrosis were discovered in the myocardial interstitium of the model group rats, and this myocardial fibrosis was dose-dependently reduced by treatment with ASP (Figure 2(b)). Then, we have taken the immunofluorescence assay, RT-qPCR, and western blot analyses to detect the change of cell matrix-related gene expression in the heart tissues. The result of the immunofluorescence assay showed that *α*-SMA and TGF-*β*1 were overexpressed in the model group rats, while the expression levels were decreased in the rats treated with APS, with the tendency along with the increase in the ASP dose (Figure 2(c)). Meanwhile, the data of RT-qPCR and western blot analyses revealed that both of the mRNA and protein expression levels of collagen I, *α*-SMA, fibronectin, and vimentin were increased in the HHD rats, when compared with the normal rats. In contrast, ASP decreased their expression levels in a dose-dependent manner in comparison with the model group rats (Figures 2(d) and 2(e)). Besides that, the measure of left ventricular mass index (LVMI) among different group rats in the 4 and 8 weeks showed that the LVMI was significantly higher in HHD rats compared with the normal rats, and ASP significantly decreased the change of LVMI in a dose-dependent manner (Figure 2(f)). Taken together, we found that ASP could inhibit cardiac fibrosis induced by hypertensive in rats.

### 3.3. Angelica sinensis Polysaccharide Suppresses Cardiomyocyte Apoptosis in Hypertensive Rats

Next, to further evaluate the alleviated effects of ASP on cardiac dysfunction induced by hypertension in rats, we evaluated the myocardial apoptosis by TUNEL staining assays and quantifying the expression of key apoptotic components. The tissue slices analyzed by TUNEL staining assays showed significantly myocardial apoptosis in HHD rats in comparison with the normal rats, and ASP significantly decreased the myocardial apoptosis in a dose-dependent manner in comparison with the model group rats (Figure 3(a)). The mRNA and protein expression levels were measured by RT-qPCR and western blot analyses, which showed increased expression of Bax, cleaved caspase-3, and cleaved caspase-9 and decreased expression of Bcl-2 in HHD rats. These results indicated the occurrence of apoptosis after HFD stimulation. In contrast, different doses of ASP intervention significantly decreased the expression of Bax, cleaved caspase-3, and cleaved caspase-9, while increasing the expression of Bcl-2 compared to the model group rats (Figures 3(b) and 3(c)). All above findings indicate that ASP might suppress hypertension-induced cardiomyocyte apoptosis in rats.

### 3.4. Angelica Polysaccharide Alleviates Oxidative Stress in Cardiomyocytes of Hypertensive Rats

Finally, we assessed the protective efficacy of ASP against hypertension-induced oxidative stress in rat cardiomyocytes. The detection of the oxidative stress marker showed that H_2_O_2_ and MDA levels were significantly elevated in the HHD rats in comparison with the normal rats, while the activity of GSH-Px and SOD was significantly decreased. However, these variations were alleviated by ASP therapy, and all of the alleviation was in an ASP dose-dependent manner (Figure 4(a)). Besides that, the HHD rats were measured with significantly higher level of ROS in the left ventricle compared to the normal rats. And ASP significantly decreased the level of ROS in a dose-dependent manner in comparison with the model group rats (Figure 4(b)). The above findings demonstrated that ASP alleviated hypertension-induced oxidative stress in rats.

## 4. Discussion

Cardiovascular diseases, especially hypertrophy heart disease, are the leading cause of mortality and morbidity in the global world. Hypertensive heart disease which can lead to death is one of the most common complications in hypertensive patients [2]. A previous study has shown that, during the process of hypertension, the high blood pressure could increase the workload on the heart and change the structural and functional feature of the myocardium. These changes include cardiomyocyte apoptosis, oxidative stress of cardiac myocytes, and hypertrophy of the left ventricle. All of these can progress to heart failure [3]. Therefore, the treatments for preventing hypertensive heart disease via improving ventricular remodeling and suppressing cardiomyocyte apoptosis may be important strategies to the reduction of hypertensive patients' morbidity and mortality [15, 16].

It is known that the decrease in EF and FS indicates that spontaneously hypertensive rats (SHRs) exhibited ventricular remodeling and dysfunction [8]. In this study, we established an HFD-induced HHD rat model according to the previous report [14]. The detection of EF and FS decrease in HHD rats indicated ventricular remodeling and dysfunction. Then, we explored the potential effects of ASP extracted from the Lixinshui prescription on cardiac function in HHD rats. After administration of a low, middle, or high dose of ASP, the EF and FS were increased in HHD rats. Besides that, the measurement of left ventricle function indicated that ASP could decrease the LVEDD, LVESD, LVEDV, and LVESV in HHD rats. As it is known, the LVEDD and LVESD were increased in chronic heart failure rats [2]. The data of our study implicated the role of ASP in improving HFD-induced hypertensive rat heart function and preventing hypertensive heart disease.

Fibrosis is generally considered a major factor of remodeling and stiffening [17]. Myocardial fibrosis (MF) was an important pathophysiological process in cardiovascular disease, often leading to malignant arrhythmia, heart failure, and even sudden death [18]. The pathological basis of myocardial fibrosis includes proliferation of cardiac fibroblasts (CFs) and excessive deposition of extracellular matrix (ECM) components [19]. In the present study, the detection of H&E- and Masson's trichrome-stained tissue showed disorderly arranged myocardial cells and significantly thickened muscle fibers in the myocardial interstitium of the HHD rats. Meanwhile, ASP significantly alleviated the disorderly arrangement of muscle fibers in a dose-dependent manner.

As previous studies reported, increased *α*-SMA and collagen I expression levels are important markers of liver fibrosis [20]. TGF-*β*1, as a major fibrogenic factor, could promote the epithelial-mesenchymal transition (EMT) and lung fibroblast-to-myofibroblast transdifferentiation [21]. Fibronectin and vimentin are fibroblastic markers and play an important role in the process of EMT and tumorigenesis in colorectal carcinoma [22]. ICG-001 has been reported to attenuate myocardial fibrosis and inhibited alpha-smooth muscle actin, fibronectin, and collagen I expression in Ang II-induced cardiac hypertrophy rats [23]. Our study demonstrated that ASP reversed the overexpression of *α*-SMA, TGF-*β*1, collagen I, fibronectin, and vimentin in the rats fed with an HFD. In addition, we examined the apoptosis of left ventricular cardiomyocytes using TUNEL staining. The results showed that the number of positive cells got increased in the HFD group while which got decreased in the ASP-treated groups. Besides that, the result of RT-qPCR and western blot analyses revealed that different doses of ASP intervention decreased the expression of Bax, cleaved caspase-3, and cleaved caspase-9, while increasing the expression of Bcl-2. All of these results indicate that ASP improved left ventricular remodeling by suppressing cardiac fibrosis and inhibiting cardiomyocyte apoptosis.

Oxidative stress is characteristically associated with vascular dysfunction and cardiovascular remodeling [24]. The imbalance between oxidants and antioxidants in favor of the oxidants caused ROS excessive accumulation [25]. Physiologically, ROS stimulates the proliferation of cardiac fibroblasts leading to ECM remodeling [26]. In this study, we found that ASP could decrease the level of H_2_O_2_ and MDA and elevated the activity of GSH-Px and SOD in the HHD rats. Meanwhile, ASP could decrease the level of ROS in a dose-dependent manner. Taken together, these results demonstrated that ASP may inhibit cardiac fibrosis and suppress cardiomyocyte apoptosis by alleviating oxidative stress.

Regrettably, our experiment did not conduct a verification study on the function of ASP in other kinds of hypertension models. Our results demonstrated the effect of ASP on preventing hypertensive heart disease *in vivo*. In the future research, we will focus on the underlying mechanisms of ASP on hypertensive heart disease prevention, as ROS is also involved in a variety of factors to induce cardiovascular disease.

## 5. Conclusions

ASP extracted from the Lixinshui prescription prevents hypertensive heart disease by improving cardiac function, inhibiting cardiac fibrosis, suppressing cardiomyocyte apoptosis, and alleviating oxidative stress. Our findings demonstrate that ASP, as an active component of the Lixinshui prescription, is an excellent candidate for hypertension heart disease. These findings will facilitate the development of traditional Chinese herbs in modern medicine.

## Figures and Tables

**Figure 1:** ASP treatment alleviates cardiac function *in vivo*. The rats were induced to hypertensive heart disease (HHD) rats by high-fat diet (HFD) randomly divided into three doses of ASP-treated groups and a vehicle-treated group. Meanwhile, the standard diet-fed rats were treated with distill water as a normal control group. (a) The body weight was measured during the experimental process. (b) Left ventricle function was measured including left ventricle end-diastolic volume (LVEDV), left ventricle end-diastolic diameter (LVEDD), left ventricle end-systolic diameter (LVESD) and left ventricular end-systolic volume (LVESV), left ventricular ejection fraction (EF), and left ventricular short axis shortening rate (FS). Three independent experiments were performed. The graph shows the mean ± SD calculated for at least three experiments. ^∗^^or #^*p* < 0.05, ^∗∗^^or ##^*p* < 0.01.

**Figure 2:** ASP treatment inhibits cardiac fibrosis *in vivo*. H&E (a) and Masson's (b) staining assays were performed to demonstrate the effects of ASP on cardiac fibrosis of rat left ventricular tissues. (c) Immunohistochemical analysis of *α*-SMA and TGF-*β*1 protein levels in rat left ventricular tissues. (d) LVMI was measured in the different sample groups. The expression levels of collagen I, *α*-SMA, fibronectin, and vimentin were evaluated by performing RT-qPCR (e) and western blot assays (f) in the different sample groups. Protein expression levels relative to *β*-actin levels are shown. Three independent experiments were performed. The graph shows the mean ± SD calculated for at least three experiments. ^∗^^or #^*p* < 0.05, ^∗∗^^or ##^*p* < 0.01.

**Figure 3:** ASP treatment inhibits the apoptosis of cardiomyocytes *in vivo*. TUNEL staining assays were performed to demonstrate the apoptosis of cardiac myocytes in rat left ventricular tissues. The expression levels of Bax, Bcl-2, cleaved caspase-3, and cleaved caspase-9 were evaluated by performing RT-qPCR (b) and western blot assay (c) in the different sample groups. Protein expression levels relative to *β*-actin levels are shown. Three independent experiments were performed. The graph shows the mean ± SD calculated for at least three experiments. ^∗^^or #^*p* < 0.05, ^∗∗^^or ##^*p* < 0.01, and ^∗∗∗^^or ###^*p* < 0.001.

**Figure 4:** ASP treatment alleviates oxidative stress of cardiomyocytes *in vivo*. Five oxidative and antioxidative parameters including the activity of GSH-Px and SOD, the level of ROS, endogenous hydrogen peroxide (H_2_O_2_), and MDA were determined by the corresponding measure in the left ventricle tissues from different group rats. Three independent experiments were performed. The graph shows the mean ± SD calculated for at least three experiments. ^∗^^or #^*p* < 0.05, ^∗∗^^or ##^*p* < 0.01.

**Table 1:** The primer sequences.

Gene name	Direction	Primer sequence (5′‐3′)
*β*-Actin	Forward	ATGACGATATCGCTGCGCTC
	Reverse	CCCATACCCACCATCACACC
Collagen I	Forward	GACATGTTCAGCTTTGTGGACCTC
	Reverse	GGGACCCTTAGGCCATTGTGTA
*α*-SMA	Forward	CCGAATGCAGAAGGAGATCA
	Reverse	GTGGACAGAGAGGCCAGGAT
Fibronectin	Forward	CCTACGGCCACTGTGTCACC
	Reverse	AGTCTGGGTCACGGCTGTCT
Vimentin	Forward	AATGACCGCTTCGCCAAC
	Reverse	CCGCATCTCCTCCTCGTAG
BAX	Forward	TGGCGATGAACTGGACAACA
	Reverse	TAGAAAAGGGCAACCACCCG
Bcl-2	Forward	CTGGTGGACAACATCGCTCT
	Reverse	GCATGCTGGGGCCATATAGT
Cleaved caspase-3	Forward	TGGAAGCGAATCAATGGACTCTGG
	Reverse	CCAGACCGAGATGTCATTCCAGTG
Cleaved caspase-9	Forward	CTGCTGCGTGGTGGTCATTCTC
	Reverse	CACAATCTTCTCGACCGACACAGG

## Data Availability

All data generated or analyzed during this study are included in this published article.
